# Influencing Factors and Prevention of Sepsis or Acute Kidney Injury in 85 Patients with Severe Trauma

**DOI:** 10.1155/2021/5754114

**Published:** 2021-11-03

**Authors:** Hong Zhang, Dan Chen, Lihua Wang, Bing Li

**Affiliations:** ^1^Nephrology Department, Taizhou Hospital of Zhejiang Province, Linhai, Zhejiang 317000, China; ^2^Special Ward, Taizhou Hospital of Zhejiang Province, Linhai, Zhejiang 317000, China; ^3^Emergency Department, Taizhou Hospital of Zhejiang Province, Linhai, Zhejiang 317000, China

## Abstract

Severe trauma can cause systemic reactions, leading to massive bleeding, shock, asphyxia, and disturbance of consciousness. At the same time, patients with severe trauma are at high risk of sepsis and acute renal injury. The occurrence of complications will increase the difficulty of clinical treatment, improve the mortality rate, and bring heavy physical and mental burdens and economic pressure to patients and their families. It is of great clinical significance to understand the high risk factors of sepsis and AKI and actively formulate prevention and treatment measures. In this study, the clinical data of 85 patients with severe trauma were analyzed by univariate and multivariate logistic regression to identify the risk factors leading to sepsis or AKI and analyze the prevention and treatment strategies. The results showed that multiple injuries, APACHE II score on admission, SOFA score on admission, and mechanical ventilation were independent influencing factors of sepsis in patients with severe trauma, while hemorrhagic shock, APACHE II score on admission, CRRT, and sepsis were independent influencing factors of AKI in patients with severe trauma. Severe trauma patients complicated with sepsis or AKI will increase the risk of death. In the course of treatment, prevention and intervention should be given as far as possible to reduce the incidence of complications.

## 1. Introduction

Sepsis and acute kidney injury (AKI) are common complications after severe trauma. Sepsis is prone to shock and multiple organ failure, while AKI is prone to hyperkalemia and volume overload, both of which will significantly increase the risk of death and pose a serious threat to the life and health of patients [1]. In recent years, clinical studies have mainly focused on the pathophysiological process of sepsis or AKI after trauma. Although monitoring and treatment techniques have been innovated and developed, the prognosis of sepsis and AKI has not been significantly improved and is still a risk factor for death in patients with severe trauma [2, 3]. It is of great significance to further understand the factors related to the occurrence of complications and carry out active prevention and treatment according to them. The emergency surgery department of our hospital has been treating many patients for many years and has accumulated rich clinical case data and experience. Therefore, the clinical data of 85 severe trauma patients were collected in this study, and the relevant factors affecting sepsis or AKI were discussed after summary and analysis. Based on this, the prevention and treatment strategies were discussed to provide a theoretical basis for clinical prevention and early diagnosis.

## 2. Methods

### 2.1. General Information

The clinical data of 85 patients with severe trauma admitted to our hospital from May 2014 to May 2019 were retrospectively analyzed, including 62 males and 23 females, aged from 21 to 58 years old, with an average age of 43.21 ± 11.68 years. There were 34 patients complicated with sepsis, including 23 males and 11 females, with an average age of 45.12 ± 6.14 years, and 51 patients without sepsis, including 39 males and 12 females, with an average age of 44.97 ± 6.23 years. And there were 27 patients with AKI, including 18 males and 9 females, with an average age of 44.83 ± 9.57 years, and 58 patients without AKI, including 44 males and 14 females, with an average age of 44.32 ± 10.29 years. There was no statistical difference in general data between patients complicated with sepsis and those without sepsis and between patients complicated with AKI and those without AKI, which indicates comparability (*P* > 0.05).

### 2.2. Inclusion Criteria

The inclusion criteria were defined as follows: (i) patients with a history of trauma and an injury severity score (ISS) ≥ 16; (ii) patients complicated with sepsis are in accordance with the relevant diagnostic criteria of “Chinese Guidelines for the Treatment of Severe Sepsis/Septic Shock” [4], specifically with body temperature >38.5°C, heart rate >90 beats/min, and serum white blood cell count > 10.8 × 109/L or <4.0 × 109/L; and the number of bacteria per gram of subeschar tissue was ≥1 × 105, and the biopsy showed bacterial invasion to biopsy tissues, with sepsis-related clinical manifestations; (iii) patients complicated with AKI meet the relevant diagnostic criteria in the Guide to Clinical Practice of KDIGO for Acute Kidney Injury [5]. The renal function decreased rapidly within 48 h, the absolute value of serum creatinine increased ≥26.5 *μ*mol/L or increased ≥50% than the basal value within 7d, and (or) urine volume <0.5 ml/ (kg·h) lasted for more than 6 h.

### 2.3. Exclusion Criteria

The exclusion criteria were defined as follows: (i) patients with the acute or chronic infection prior to the occurrence of trauma, (ii) patients with past severe circulatory and immune system diseases, (iii) patients with past liver and kidney insufficiency, and (iv) patients who have incomplete or inaccurate clinical data.

### 2.4. Research Methods

The clinical data of all patients were collected, including the age, gender, type of trauma, multiple trauma, acute physiology and chronic health evaluation II (APACHE II) score on admission, sequential organ failure assessment (SOFA) score on admission, ISS on admission, diabetes mellitus, hypertension, mechanical ventilation, surgical treatment, massive blood transfusion, hemorrhagic shock, and continuous renal replacement therapy (CRRT).

The APACHE II score included acute physiology score, age score, and chronic health status score. APACHE II score was calculated according to clinical data and laboratory test indexes within 24 hours after admission. The theoretical maximum score was 71, and a higher score indicated a more critical condition [6].

The SOFA scores include seven organ systems: respiratory, circulatory, kidney, coagulation, nervous, liver, and gastrointestinal. The total score ranges from 0 to 28, with a higher score indicating a more serious condition [7].

The ISS divides the injury sites into six parts: head and neck, face, chest, abdomen and pelvis, limbs and pelvis, and body surface. The degree of trauma in each part is divided into six levels: mild, moderate, severe but not life-threatening, severe but life-threatening but survivable, extremely severe, and unable to rescue success, and the corresponding score is 1, 2, 3, 4, 5, and 6. The effective range of SS score was 1–75 points. The higher the score was, the more serious the injury would be [6].

### 2.5. Statistical Methods

All data were processed with SPSS 22.0 statistical software, and GraphPad prism 8 was used to make statistical graphs. Measurement data are expressed as mean ± standard deviation ($\bar{x}$ ± *s*); independent sample *t*-test is used for comparison between groups; count data is expressed as [*n*(%)]; and chi-square (*𝒳*^2^) test is performed. Univariate analysis and multivariate logistic regression model were used to analyze the influencing factors of sepsis or AKI in severe trauma patients. The difference is statistically significant when *P* < 0.05.

## 3. Results

### 3.1. Univariate Analysis of Sepsis in Severe Trauma Patients

Univariate analysis showed that there were no differences in age, gender, diabetes, hypertension, hemorrhagic shock, and CRRT between patients with and without sepsis (*P* > 0.05). However, there were statistically significant differences in the type of trauma, multiple injuries, APACHE II score on admission, SOFA score on admission, ISS on admission, mechanical ventilation, surgical treatment, and massive blood transfusion between patients complicated with and without sepsis (*P* < 0.05; Table 1).

### 3.2. Multifactorial Analysis of Sepsis in Patients with Severe Trauma

Patients with sepsis were taken as dependent variables, and factors with significant differences in Table 1 were included in the logistic regression model as independent variables. The assignment of dependent variables and independent variables is shown in Table 2.

Logistic regression analysis showed that multiple injuries, APACHE II score on admission, SOFA score on admission, and mechanical ventilation were independent risk factors for sepsis in severe trauma patients (*P* < 0.05; Table 3).

### 3.3. Univariate Analysis of AKI in Severe Trauma Patients

There was no difference in age, gender, type of trauma, diabetes, hypertension, mechanical ventilation, surgical treatment, and massive blood transfusion between patients with and without AKI. However, there were statistically significant differences in multiple injuries, APACHE II score on admission, SOFA score on admission, ISS on admission, hemorrhagic shock, CRRT, and sepsis in patients with and without AKI (*P* < 0.05; Table 4).

### 3.4. Multifactorial Analysis of AKI in Patients with Severe Trauma

Patients with AKI were taken as dependent variables, and factors with significant differences in Table 4 were included in the logistic regression model as independent variables. The assignment of dependent variables and independent variables is shown in Table 5.

Logistic regression analysis showed that hemorrhagic shock, APACHE II score on admission, CRRT, and sepsis were all independent risk factors for AKI in severe trauma patients (*P* < 0.05; Table 6).

## 4. Discussion

Trauma is the destruction of human tissues or organs caused by mechanical factors. Severe trauma can cause systemic reactions. Local manifestations include pain, swelling, tenderness in the injured area, deformity, and dysfunction when fracture and dislocation. After severe trauma, the body will have a strong physiological stress response, neuroendocrine disorder, systemic metabolic disorder, a sharp decline of organ function, and even shock. During treatment, due to long-term exposure to mucosal muscle tissue and low immune resistance, patients often have various complications. Infection is one of the main complications 48 hours after severe trauma, and it is highly likely to develop into sepsis if not properly handled. AKI is also a common complication of severe trauma patients, and its pathogenesis is relatively complex, usually related to hypovolemia caused by fluid loss, renal insufficiency, and organ shock caused by sepsis [8, 9].

AKI is also a common complication in patients with severe trauma, and its pathogenesis is complex, which is usually related to low blood volume caused by fluid loss, insufficient renal perfusion, and organ shock caused by sepsis. Our hospital has been treating trauma patients for many years, with mature clinical treatment experience [10]. It has been observed in the past that patients with severe trauma often suffer from sepsis or AKI. In this study, the association between sepsis or AKI and clinical characteristics was discussed in order to provide a reliable basis for the prevention and treatment of severe trauma complications [11]. Now, the analysis results are shared as follows.

Due to the reasons of the disease itself or the use of sedatives for anesthesia, patients are often in coma or unclear consciousness [12]. And poor blood perfusion leads to ischemia and hypoxia, wound infection, stress response, and gastrointestinal paralysis. These factors are very easy to induce acute infection or systemic inflammatory response syndrome complicated with septicemia [13]. The pathogenesis of sepsis is mainly immune abnormalities and impaired cell function. Patients with severe trauma are prone to a large number of fluid loss and immune dysfunction. The infection has also become the main contradiction after injury, and the risk of sepsis is significantly increased [13]. Sepsis is one of the causes of death in severe trauma patients, with a fatality rate of over 50%. In this study, 85 patients were collected, and 34 patients were complicated with sepsis, with the incidence rate as high as 40%, among which wound sepsis was the main one. After symptomatic support treatment, the disease of most patients has been effectively controlled, but there are still some patients whose disease develops rapidly and evolves into full-blown septic shock or MODS, which is a serious threat to life safety. Therefore, it is very important to guard against sepsis after injury.

Logistic regression analysis showed that multiple injuries, Apache II score on admission, SOFA score on admission, and mechanical ventilation were independent influencing factors of sepsis in patients with severe trauma (*P* < 0.05). Severe multiple injuries refers to two or more injuries caused by the same injury factor and at least one life-threatening injury. Systemic inflammatory response syndrome (SIRS) is the inevitable defense response after multiple injuries [14]. Uncontrolled inflammation should be the basic factor to induce septic shock and MODS. It is important to actively consider the prevention and treatment strategies of sepsis, SIRS, and even MODS after multiple injuries [15]. The basic treatment goal of our hospital is to reduce trauma response, shorten trauma response time, and enter the recovery period of trauma and organ function through SIRS or sepsis. Resuscitate patients with severe trauma, especially multiple injuries, were immediately given resuscitate plan after admission [16]. At the same time, the biochemical and molecular indicators were strictly detected, and infection lesions and secondary infection lesions were actively sought and cleared to block the process of sepsis [17].

APACHE II score is the most widely used and authoritative critical illness evaluation system in severe patients, which can objectively evaluate the severity of disease [18]. The higher the APACHE II score is, the more severe the disease is and the worse the prognosis is. Assessment of APACHE II in the emergency room or at admission to ICU is more significant [19]. Systemic multiple organ failure is the result of the occurrence and development of sepsis. And the SOFA score reflects the severity of the disease by evaluating organ function status, which is closely related to the prognosis of sepsis. The higher the score is, the more serious the organ function decline is. Our hospital attaches great importance to the assessment of APACHE II and SOFA in severe trauma patients at the beginning of admission so as to be alert to the potential risk of organ dysfunction caused by sepsis and timely provide organ support therapy.

Patients with severe trauma often need early respiratory support and mechanical ventilation when necessary [20]. Mechanical ventilation can damage airway mucosa and other tissues to a certain extent, resulting in congestion, swelling, and inflammatory exudation. In the case of low immune function, airway inflammation can induce SIRS and sepsis. For trauma patients in our hospital, the airway secretions were cultured regularly; the antibiotics were given symptomatic prevention and treatment; and the drugs were given directly to the respiratory tract when necessary [21, 22]. Meanwhile, nutrition therapy and other systemic supportive therapies have to be strengthened to improve immunity.

The incidence of AKI in patients with severe trauma can be as high as 30%, which significantly increases the risk of death. M. Eriksson et al. pointed out that AKI was a common complication in ICU hospitalized trauma patients with a high mortality rate. Diabetes, male sex, and severe injury are risk factors [23]. Patients with severe trauma suffered systemic damage and a variety of physiological functions were affected and abnormal, leading to insignificant early symptoms of AKI. So it is of great significance to explore the related influencing factors for the occurrence of AKI. In our study, 27 cases were complicated with AKI, with an incidence of 31.76%. According to the case data, the etiology of AKI is complex, which is usually the result of multiple factors. This study conducted statistical analysis on severe trauma patients complicated with AKI.

Logistics regression analysis showed that hemorrhagic shock, APACHE II score on admission, CRRT, and sepsis were independent influencing factors of AKI in patients with severe trauma (*P* < 0.05). Severe trauma patients complicated with shock usually result in multiple organ dysfunction. After the occurrence of hemorrhagic shock, the kidney is severely ischemic and hypoxic, which leads to energy metabolism disorder and further leads to the incomplete and impaired function of related tissue cells in the kidney. In addition, a large number of oxygen free radicals produced during ischemia-reperfusion injury can cause renal damage. For patients with hemorrhagic shock, our hospital corrected shock and hypoxia as soon as possible, shortened renal ischemia time, and maintained good internal blood perfusion so as to avoid and reduce renal damage.

The APACHE II score and SOFA score have been widely used in the comprehensive evaluation of severe trauma. APACHE II score can quickly evaluate the basic physiological function of patients. Therefore, with high APACHE II scores, patients have severe circulatory insufficiency and renal hypoperfusion, which can trigger AkI [24]. For patients with large trauma, fluid resuscitation was given in our hospital as soon as possible in order to restore effective circulating blood volume as soon as possible and ensure normal blood perfusion.

Our hospital summarized clinical experience and found that after severe trauma patients went through the shock period, damaged muscle fibers were dissolved, and a large amount of intracellular components such as myoglobin and denature protein were released into the blood, which stimulated inflammation and oxidative stress. At this time, the implementation of CRRT helps remove excessive intracellular components and inflammatory mediators in the body so as to avoid muscle lysis products and toxins blocking renal tubules and causing renal vascular tissue damage. CRRT indicates that the metabolic rate of renal function in patients is not enough to remove myoglobin and other components in a timely manner [25]. Therefore, the author believes that patients undergoing clinical CRRT are more likely to develop AKI. Sepsis is a key risk factor for AKI, and its pathophysiological process is the result of multiple factors. On the one hand, sepsis leads to systemic vascular dysfunction, high flow, and low pressure state, and renal vascular flow deficiency necrosis, leading to AKI [26]. On the other hand, when sepsis occurs, a large number of inflammatory mediators are released into the blood, leading to vascular endothelial injury and inflammatory response of renal artery and other vascular tissues, which is the main pathogenesis of sudden decline in renal function [27]. In this study, 18 of the 27 patients complicated with AKI were complicated with sepsis. Therefore, monitoring the signs of infection in patients with severe trauma at any time and early preventive use of antibiotics according to the results of pathogen culture and drug sensitivity are not only conducive to the prevention and treatment of sepsis but also to the reduction of the risk of AKI.

In summary, the multiple injuries, APACHE II score on admission, SOFA score on admission, and mechanical ventilation were independent influencing factors of sepsis in patients with severe trauma, while hemorrhagic shock, APACHE II score on admission, CRRT, and sepsis were independent influencing factors of AKI in patients with severe trauma. Severe trauma patients complicated with sepsis or AKI will increase the risk of death. In the course of treatment, prevention and intervention should be given as far as possible to reduce the incidence of complications. The deficiency of this study lies in the small sample size, which can be expanded in the future, and the related mechanisms of sepsis and AKI after severe trauma can be revealed through multiple research directions.

## Figures and Tables

**Table 1:** Univariate analysis of sepsis in severe trauma patients.

Clinical information	Concurrent sepsis group (*n* = 34)	Uncomplicated sepsis group (*n* = 51)	*𝒳* ^2^/*t*	*P*
Age	45.12 ± 6.14	44.97 ± 6.23	0.109	0.913

*Gender*				
Male	23 (67.60)	39 (76.47)	0.805	0.370
Female	11 (32.40)	12 (23.53)		

*Type of trauma*				
Open	24 (70.60)	13 (25.49)	16.879	≤0.001
Close	10 (29.40)	38 (74.51)		

*Multiple trauma*				
No	11 (32.40)	40 (78.43)	18.047	≤0.001
Yes	23 (67.60)	11 (21.57)		

APACHE II score on admission	51.59 ± 10.43	43.66 ± 8.31	3.888	≤0.001
SOFA score on admission	18.34 ± 2.58	14.11 ± 1.90	8.701	≤0.001
ISS on admission	30.74 ± 3.81	23.15 ± 2.19	11.649	≤0.001

*Diabetes*				
No	13 (38.20)	22 (43.14)	0.202	0.653
Yes	21 (61.80)	29 (56.86)		

*Hypertension*				
No	20 (58.80)	25 (49.02)	0.120	0.729
Yes	24 (70.60)	26 (50.98)		

*Mechanical ventilation*				
No	9 (26.50)	37 (72.55)	17.444	≤0.001
Yes	25 (73.50)	14 (27.45)		

*Surgical treatment*				
No	10 (29.40)	35 (68.63)	12.593	≤0.001
Yes	24 (70.60)	16 (31.37)		

*Massive blood transfusion*				
No	13 (38.20)	39 (76.47)	12.557	≤0.001
Yes	21 (61.80)	12 (23.53)		

*Hemorrhagic shock*				
No	16 (47.10)	23 (45.10)	0.032	0.859
Yes	18 (52.90)	28 (54.90)		

*CRRT*				
No	20 (58.80)	29 (58.86)	0.032	0.858
Yes	14 (41.20)	22 (43.14)		

**Table 2:** Assignment for multivariate analysis of severe trauma patients with complicated sepsis.

Variable	Assignment
*Dependent variable*	
Concurrent sepsis	No = 0, yes = 1
*Independent variables*	
Type of trauma	Close = 0, open = 1
Multiple injuries	No = 0, yes = 1
APACHE II score on admission	Enter as the actual score
SOFA score on admission	Enter as the actual score
ISS on admission	Enter as the actual score
Mechanical ventilation	No = 0, yes = 1
Surgical treatment	No = 0, yes = 1
Massive blood transfusion	No = 0, yes = 1

**Table 3:** Multifactorial analysis of sepsis in patients with severe trauma.

Factors	*β*	SE	Wald	*P*	OR	95% CI
Type of trauma	0.856	0.361	2.986	0.426	0.563	0.154∼1.127
Multiple injuries	1.625	0.776	4.385	0.021	1.254	0.820∼2.288
APACHE II score on admission	0.581	0.407	2.038	0.236	1.086	0.922∼1.348
SOFA score on admission	1.187	0.491	5.844	0.045	1.170	0.934∼2.424
ISS on admission	1.241	0.523	5.630	0.040	1.192	0.946∼2.443
Type of trauma	0.819	0.377	3.134	0.469	0.646	0.469∼1.156
Mechanical ventilation	1.589	0.364	4.759	0.030	1.856	0.795∼2.658
Surgical treatment	0.656	0.395	3.758	0.206	0.952	0.776∼1.298
Massive blood transfusion	0.874	0.541	3.571	0.135	0.859	0.859∼2.481

**Table 4:** Univariate analysis of AKI in severe trauma patients.

Clinical information	Concurrent AKI group (*n* = 27)	Uncomplicated AKI group (*n* = 58)	*𝒳* ^2^/*t*	*P*
Age	44.83 ± 9.57	44.32 ± 10.29		

*Gender*				
Male	18 (66.67)	44 (75.86)	0.789	0.374
Female	9 (33.33)	14 (24.14)		

*Type of trauma*				
Open	10 (37.04)	27 (46.55)	0.679	0.410
Close	17 (62.96)	31 (53.45)		

*Multiple trauma*				
No	3 (11.11)	48 (82.76)	39.406	≤0.001
Yes	24 (88.89)	10 (17.24)		

*APACHE II score on admission*	50.95 ± 11.24	44.18 ± 7.52	3.267	≤0.001
SOFA score on admission	19.32 ± 1.79	15.02 ± 1.28	12.597	≤0.001
ISS on admission	31.66 ± 2.57	24.76 ± 2.08	13.144	≤0.001

*Diabetes*				
No	10 (37.04)	25 (43.10)	0.280	0.597
Yes	17 (62.96)	33 (56.90)		

*Hypertension*				
No	15 (55.56)	30 (51.72)	0.109	0.742
Yes	12 (44.44)	28 (48.28)		

*Mechanical ventilation*				
No	16 (59.26)	30 (51.72)	0.421	0.516
Yes	11 (40.74)	28 (48.28)		

*Surgical treatment*				
No	13 (48.15)	32 (55.17)	0.356	0.546
Yes	14 (51.85)	26 (44.83)		

*Massive blood transfusion*				
No	19 (70.37)	33 (56.90)	1.408	0.235
Yes	8 (29.63)	25 (43.10)		

*Hemorrhagic shock*				
No	7 (25.93)	32 (55.17)	6.347	0.012
Yes	20 (74.07)	26 (44.83)		

*CRRT*				
No	8 (29.63)	41 (70.69)	12.722	≤0.001
Yes	19 (70.37)	17 (29.31)		

*Sepsis*				
No	6 (22.22)	45 (77.59)	23.530	≤0.001
Yes	21 (77.78)	13 (22.41)		

**Table 5:** Assignment for multivariate analysis of concurrent AKI in patients with severe trauma.

Variable	Assignment
*Dependent variable*	
Concurrent AKI	No = 0, yes = 1
*Independent variables*	
Hemorrhagic shock	Close = 0, open = 1
SOFA score on admission	Enter as the actual score
APACHE II score on admission	Enter as the actual score
ISS on admission	Enter as the actual score
Multiple injuries	No = 0, yes = 1
CRRT	No = 0, yes = 1
Sepsis	No = 0, yes = 1

**Table 6:** Multifactorial analysis of AKI in patients with severe trauma.

Factors	*β*	SE	Wald	*P*	OR	95% CI
Hemorrhagic shock	1.637	0.536	9.328	0.008	2.450	1.133∼12.891
SOFA score on admission	0.984	0.652	2.278	0.065	1.053	0.922∼2.491
APACHE II score on admission	1.275	0.667	3.654	0.024	2.197	1.825∼3.089
ISS on admission	0.258	0.204	1.600	0.297	0.859	0.653∼1.341
Multiple injuries	0.325	0.239	1.849	0.143	0.916	0.745∼1.292
CRRT	1.686	0.852	3.916	0.011	1.254	0.951∼2.578
Sepsis	2.364	1.067	4.908	0.004	6.420	1.394∼25.325

## Data Availability

The data used during the current study are available from the corresponding author upon request.
